# Predicting Breast Cancer Leveraging Supervised Machine Learning Techniques

**DOI:** 10.1155/2022/5869529

**Published:** 2022-08-16

**Authors:** Sanam Aamir, Aqsa Rahim, Zain Aamir, Saadullah Farooq Abbasi, Muhammad Shahbaz Khan, Majed Alhaisoni, Muhammad Attique Khan, Khyber Khan, Jawad Ahmad

**Affiliations:** ^1^Department of Computer and Software Engineering, National University of Sciences and Technology, Islamabad 44000, Pakistan; ^2^Faculty of Science and Technology, University of Tromsø, Tromso, Norway; ^3^Department of Data Science, National University of Computer and Emerging Sciences, Islamabad 44000, Pakistan; ^4^Department of Electrical Engineering, National University of Technology, Islamabad 44000, Pakistan; ^5^Department of Electrical Engineering, HITEC University, Taxila 47080, Pakistan; ^6^Computer Sciences Department, College of Computer and Information Sciences, Princess Nourah bint Abdulrahman University, Riyadh 11671, Saudi Arabia; ^7^Department of Computer Science, HITEC University, Taxila, Pakistan; ^8^Department of Computer Science, Khurasan University, Jalalabad, Afghanistan; ^9^School of Computing, Edinburgh Napier University, Edinburgh EH10 5DT, UK

## Abstract

Breast cancer is one of the leading causes of increasing deaths in women worldwide. The complex nature (microcalcification and masses) of breast cancer cells makes it quite difficult for radiologists to diagnose it properly. Subsequently, various computer-aided diagnosis (CAD) systems have previously been developed and are being used to aid radiologists in the diagnosis of cancer cells. However, due to intrinsic risks associated with the delayed and/or incorrect diagnosis, it is indispensable to improve the developed diagnostic systems. In this regard, machine learning has recently been playing a potential role in the early and precise detection of breast cancer. This paper presents a new machine learning-based framework that utilizes the Random Forest, Gradient Boosting, Support Vector Machine, Artificial Neural Network, and Multilayer Perception approaches to efficiently predict breast cancer from the patient data. For this purpose, the Wisconsin Diagnostic Breast Cancer (WDBC) dataset has been utilized and classified using a hybrid Multilayer Perceptron Model (MLP) and 5-fold cross-validation framework as a working prototype. For the improved classification, a connection-based feature selection technique has been used that also eliminates the recursive features. The proposed framework has been validated on two separate datasets, i.e., the Wisconsin Prognostic dataset (WPBC) and Wisconsin Original Breast Cancer (WOBC) datasets. The results demonstrate improved accuracy of 99.12% due to efficient data preprocessing and feature selection applied to the input data.

## 1. Introduction

In recent years, humans have become more prone to various types of cancer than they have ever been. Cancer is a leading cause of death worldwide and is considered to be responsible for one out of every six fatalities [1]. The most common type of cancer in terms of new cases is breast cancer. Breast cancer alone claimed the lives of around 40,920 women in 2018 [1, 2]. According to the World Health Organization (WHO), around 2.90 million women are diagnosed with breast cancer every year [3]. The term cancer refers to more than 100 diseases that affect different regions of the human body. To understand the beginning of cancer, an insight into the normal cell division is required. Cells are the fundamental units that undergo programmed cell death (apoptosis) and proliferate (via mitosis) to regenerate. But sometimes, environmental and genetic factors interfere with the programmed process of division or death and begin to grow uncontrollably resulting in a mass of cells called a tumor. The tumor can be cancerous and has the ability to metastasize to other parts of the body and cause pathology [3]. A benign tumor, on the other hand, means that the tumor is not malignant. For the treatment of any type of cancer, early detection is an essential factor. Therefore, it is important to exploit different diagnostic methods for the automated detection of cancer. Breast cancer is caused by the rapidly proliferating cells that develop breast lumps [4, 5]. As per the reports of the World Health Organization (WHO), breast cancer is among the top-ranked reasons for fatalities in women. Hence, it is critical that in addition to the diagnosis, the treatment of breast cancer is equally important at the early stages. The diagnosis of breast cancer can be made possible because of physiological changes in the breast; therefore, monitoring and screening of breast cancer on a regular basis are important and can help in the early diagnosis of the disease.

Machine learning (ML) methods have extensively been utilized over the last few decades to develop various predictive models which are capable of effective decision making. Similarly, the use of machine learning can drastically improve the automated decision-making process and can prove to be an excellent aid to medical practitioners in the early and precise detection of breast cancer. ML techniques can effectively be utilized to identify various patterns in a dataset and, hence, can predict the type of cancer (either malignant or benign). For the automated detection of breast cancer, various important parameters, i.e., marginal adhesion, clump thickness, and uniformity of cell shape or size (bland chromatin, the normality of nuclei, single epithelial cell size, and mitosis), are extracted from breast cancer mammography (X-ray pictures). In addition to these, some other factors, such as age, number of previous biopsies, and the number of the first-degree relatives having breast cancer, can also be used to predict the occurrence and repetition of breast cancer. Furthermore, for the prediction of breast cancer using ML techniques, the utilized data may also include parameters from the blood analyses reports such as BMI, age, HOMA, glucose, and leptin. Moreover, the nonpathological data, such as ethnicity, pregnancy history, nursing history, obesity, radiation or carcinogenic chemical exposure to the face or chest in the early 30s or before, poor levels of vitamin D, sedentary lifestyle, and irregular menstrual history, can also be helpful in the prediction and diagnosis of breast cancer using ML approaches.

By carefully selecting features and manipulating data, we present a unique approach for the diagnostic prediction of breast cancer in our work. We used the WDBC dataset to diagnose features [6]. The study is aimed at predicting the tumor with high accuracy even with a reduced set of attributes. Existing research strictly focused on the use of traditional classification models in order to achieve accuracy. However, in our proposed solution, we have improved the overall classification process. This included handling data noise, data sampling, and applying filter-based feature selection methods for determining optimal features, followed by five classification methods for comparative analysis of the performance of different classifiers. Moreover, the performance is tested multiple times over different test-train splits to determine the best split.  Figure 1 shows the stages involved in the experiment that including the data preprocessing step, feature selection, data handling and application of classification models, and evaluation of their accuracy.

The subsequent part is organized as follows: Section 2 encompasses a literature review, leading datasets, and current problems, Section 3 of this paper discusses the solution proposed in this study, Section 4 explains the methods and experimentation process which have been used, Section 5 provides an analysis of the experimental results along with a comparative analysis with previous researches, Section 6 analyzes the results of our proposed approach on other datasets, and Section 7 discusses the conclusion and future works.

## 2. Related Work

Various researches can be found for the detection of breast cancer using different ML and neural network approaches; for example, Karabatak and Ince present a hybridized neural network-based breast cancer diagnostic system in [7]. The presented approach utilizes an association rule-based method to derive patterns from the breast cancer data. The association rules have been used to reduce the number of features, eliminating useless or less contributing features by finding relations as associations among closely related features. This technique helped in the reduction of feature space. The Wisconsin Breast Cancer dataset has been utilized for the training and testing of the presented technique. The results demonstrate the effectiveness of the presented hybridized neural network in terms of efficiency, and it also outperforms all other neural networks implemented in the study for comparison purposes [7].

Similarly, Ravdin and Clark [8] utilized a neural network to forecast a patient's chance of survival by using the prognostic data involving the time factor. A data of 1373 patients was utilized, and the neural network's prediction was also compared to that of a regression model. Moreover, Wolberg et al. [9] developed a linear diagnostic model to forecast malignant risks for nonrecurring cases and the recurring time period of diseases. This model was tested using a cross-validation approach on a dataset of 569 patients, yielding an accuracy of 97.5%. Quinlan [10] built a model for medical diagnostics and prediction by adding a Minimum Description Length (MDL) penalty to the C4.5 decision tree method, which resulted in a 94.74% accuracy. Furthermore, utilization of a large amount of data can also be found in literature; e.g., Delen et al. [11] used a big dataset of roughly 200,000 patient records. They have compared a decision tree model, i.e., C4.5, to several neural networks and linear regression models. They concluded that for large datasets, a decision tree method like C4.5 outperforms the other two, achieving an accuracy of 93.6 percent or higher.

Speaking of hybrid ML models, a hybrid model proposed by Ravi et al. [12] exhibits improved performance in terms of efficiency, because the model uses only critical features for its training. For this purpose, a combination of feature selection algorithms and fuzzy systems has been utilized. In this hybrid model, the number of rules used during the training process was minimized by using a modified threshold accepting algorithm. The model was trained on Wisconsin's Breast Cancer Classification (extracted from the UCI repository), and the Wine classification dataset. It was demonstrated that the model performs more efficiently when fewer but more relevant features are used. To further improve the performance of the model, another feature selection, and extraction method, i.e., the Principal Component Analysis (PCA) was also incorporated [12]. Similarly, Khan et al. [13] improved the learning performance by using various derivations of decision trees, including Fuzzy Decision Trees (FDT), Hybrid Decision Trees (HDT), and other related fuzzy rules to estimate the rate of recurrence for the breast cancer patients. The presented model has been trained and tested on the SEER dataset. The presented results demonstrate that the utilization of the Fuzzy Decision Tree model made the presented scheme more robust. Another hybrid approach for breast cancer classification has been proposed by Kaya and Uyar [14]. They combined the detection of diseases using rough sets and advanced machine learning algorithms. They used the breast cancer dataset acquired from the UCI repository and reported an accuracy of 98.6%.

Histopathological diagnosis serves as the gold standard for the diagnosis of malignant and benign breast cancer. However, mental anxiety and physical pain can come as a part of needle biopsy as it is invasive. Based on ultrasound images, medical image data mining methods are used in order to obtain diagnostic information of malignant and benign tumors in a noninvasive manner. The authors in [15] proposed a dictionary training-based method in order to noninvasively obtain diagnostic information. They use their method to adaptively extract different texture features for selection and classification. A data of total 128 cases were used for the study, 67 of which were malignant and 61 of which were benign resulting in a classification accuracy on 0.9070. According to 2 : 1, the dataset was divided in a random manner into training and testing sets, including 85 training sets and 43 testing sets.

The authors in [16] performed a study to analyze the effect of ultrasound technology and deep learning technology combined on the breast-conserving surgery for breast cancer. They designed a deep LDL model and introduced two models for comparison. The first was the semiautomatic segmentation algorithm RA, and the second was the segmentation model ON. They applied their designed algorithm to the breast-conserving surgery of patients suffering from breast cancer. A total of 102 female patients with early breast cancer were divided into three groups W1, W2, and W3. The W1 group contained 34 cases (ultrasound guidance based on deep learning segmentation model), the W2 group contained 34 cases (ultrasound guidance), and the W3 group contained 34 cases (palpitation guidance). The conclusion of the study suggested that the deep LDL model improved the tumor resection very effectively.

The primary attempt at computerizing medical images happened during the 1960s, which is, until now, a significant subject of research in the field of medical imaging. Recent research in AI for the medical field has given rise to computer-aided diagnostic systems. Computer-aided detection (CAD) fills in as a symptomatic guide to help the doctor's job by using accurate and noninvasive computer systems. In spite of these figures, automated detection software is not broadly utilized for the purpose of breast screening. In breast cancer imaging research, the focus has mainly been on ultrasound 2D/3D imaging combined with deep learning. The authors in [17] proposed a CAD framework for distinguishing the tumor grades of breast cancer by using US images. A total of 44 features were collected for the study. The viability of the proposed framework was checked in light of clinical data.

Various models found in the literature also report significantly high accuracies; for example, an LS-SVM classifier-based model by Polat and Güneş reports an accuracy of 98.53% and utilized 10-fold cross-validation. Another model based on an SVM classifier is proposed in [18] that demonstrates 99.02% classification accuracy even without using any cross-validation technique [18]. On the other hand, Akay et al. [19] presented an innovative and effective technique, by using combinations of swarm optimization statistical models for breast cancer detection and reported an accuracy of 98.71%. Another technique reporting a high model accuracy is proposed by Marcano-Cedeño et al. in [20]. This technique utilizes the AMMLP method by using an Artificial Neural Network over the biological metaplasticity property and reports an accuracy of 99.26%.

Similarly, there have been other cancerous and autoimmune diseases that have been worked upon such as multiple sclerosis (MS). It is an autoimmune disease that causes issues in the central nervous system up to a mild or severe extent. Like all such diseases, early detection and treatment are necessary in order to reduce the impact of the diseases. The authors in [21] propose a convolutional neural network- (CNN-) based framework (CNN) segmentation scheme for the extraction of MS lesion from a 2D brain MRI slice. They further implemented the VGG-UNet scheme in order to achieve a better MS detection. A pretrained VGG19 was considered as the encoder section. They performed their testing on 30 patient images. It was seen that their scheme provided a significantly better result in comparison to traditional UNet, VGG-SegNet, VGG-UNet and SegNet. Their experiment implemented on 2D slices of flair modality verified that this work provided with a better value of accuracy (>98%), dice (>92%), and Jaccard (>85%).

### 2.1. Limitations of Previous Frameworks

The features selected from datasets for diagnostic purposes highly impact the effectiveness and accuracy of the machine learning models [22–25]. Although various researches can be found that focus on feature selection and extraction from several popular and organized datasets, e.g., the WDBC dataset [26], it is still important to select the optimal features without changing them as it reduces the computational complexity and training time of the model and improves the accuracy to a great extent if a right subset is chosen. The typical yet significant problems like outliers, noise, unnormalized data, and high computational complexity have not been taken into consideration in previous studies. Furthermore, it is also important that the computational complexity is low. The number of features trained is linked to the computational complexity. Hence, it is important to identify the minimum number of features that will help accurately classify the tumor. In addition to feature selection, there is a dire need for new or specifically tailored model structures to improve the diagnosis.

## 3. Leading Datasets

The most commonly used datasets for breast cancer prediction include the SEER Breast Cancer (SEERBCD) [27], the Coimbra Breast Cancer (CBC) dataset [28], the Wisconsin (Prognostic) Breast Cancer (WPBC) dataset [29], the Wisconsin (Diagnostic) Breast Cancer dataset [26], the Wisconsin Original Breast Cancer (WOBC) dataset [30], and the Breast Tissue Dataset (BTD) [31]. The WPBC dataset stores data based on 30 attributes that are calculated from digital photos. The WDBC dataset is comparable to the WPBC dataset. The BTD dataset is preferred due to the inclusion of the impedance measurements of newly removed breast tissues that have been acquired at various frequencies [31]. The CBC dataset [28], on the other hand, is gathered via routine blood analysis and contains anthropometric date. This dataset contains 10 predictors in total. The predictors are quantitative, and a binary-dependent variable indicates the presence or absence of breast cancer. The SEERBCD was received in November 2017 through the National Cancer Institute's SEER program. Moreover, Dr. Wolberg's clinical cases were used to create the WOBC dataset. It contains organized chronologically data, with eight groups containing the number of instances documented between January 1989 and November 1991.

### 3.1. The WDBC Dataset

The aforementioned and some other datasets have been used in a number of research studies. However, the most used and preferred dataset is the WDBC dataset which has also been used for breast cancer diagnosis in this study. This dataset has been widely utilized because it has a large number of recorded instances (699), and the data comprises medical information of real patients, hence making the dataset an important dataset used in literature. Dr. Wolberg was the contributor to this dataset. Using a graphical computer program known as Xcyt, he obtained multiple fluid samples from patients having solid breast masses. The dataset is virtually noise-free with very few missing or outlier values. Each of the features is evaluated on a scale of 1 to 10: 1 is interpreted as being closest to benign, and 10 is interpreted as a closet to malignant. Various significant studies utilizing WDBC dataset for medical diagnosis can be found in the literature; for example, Zheng et al. [32] used the WDBC dataset and applied *K*-means and SVM algorithms for the breast cancer diagnosis. Suryachandra and Reddy [33] also utilized the WDBC dataset and compared the performance of the Bayesian belief network, DT, and SVM.

Cherkassky [34] in his study performed the analysis of WDBC using SVM with RBF and polynomial functions as kernel functions. They achieved an accuracy of 97.1%. de Bruijne [35] used a feed-forward neural network model as well as a backpropagation learning algorithm combined with momentum and variable learning rate. The study proved that the performance of multilayer neural networks is better than that of a one-layer neural network. This study also used the WDBC dataset [35]. In [36], Aryal and Paudel used the WDBC for Gradient Boosting and 10-fold cross-validation, resulting in the accuracy of 98.88% with a set of 30 features. Saygili [37] performed an analysis on this dataset recently. In his study, he used Random Forest for classification purposes and achieved an accuracy of 98.7%. He performed feature selection using Gain Ratio and used a set of 24 features and 10-fold cross-validation. Dubey et al. [38] performed on the WDBC dataset. They achieved an encouraging accuracy of 92.0%. Salama et al. [39] performed on the WDBC dataset with 30 features. They applied various different models. The best performance was demonstrated by Sequential Minimal Optimization (SMO) and 10-fold cross-validation. It resulted in an accuracy of 97.71%.  Table 1 shows a comparison of machine learning algorithms on the WDBC dataset.

## 4. The Proposed BCAD Framework

This paper presents a state-of-the-art approach to breast cancer diagnosis. The objective of the paper is to identify the most accurate machine learning model which can predict the occurrence of breast cancer based on the various patients' clinical data. In order to achieve this, we propose a hybrid method for feature selection. This method includes the use of correlation-based feature selection first, followed by the recursive feature elimination method, which helps in the reduction of the feature space. The aim is to achieve encouraging classification accuracy over a reduced number of features using the original features without changing them, as opposed to the dimensionality reduction method. Feature selection is performed in order to reduce feature space and test how much influence the feature space has over classification accuracy.

Figure 1 illustrates the BCAD framework flowcharts, which elaborate the data preprocessing, attribute selection using filter-based feature selection methods, and classification using the Multilayer Perceptron Model. As previously mentioned, the dataset utilized in this study is the Wisconsin Diagnostic Breast Cancer (WDBC) dataset which contains 569 samples. The target values (labels: M (malignant)/B (benign)) indicate that the person's tumor is malignant (cancerous) or benign (noncancerous). We have used the WDBC dataset for experimentation.

### 4.1. Data Preprocessing

The first step of the Breast Cancer Diagnostic (BCAD) framework shown in Figure 1 is data-preprocessing. In this step, the random sampling technique (which is included in Scikit Learn) creates a unique sampling distribution that is based on real data. For data visualization, the Numpy, Pandas, and Seaborn libraries are used. Large and multidimensional matrices and arrays are supported by Numpy. It also provides a mathematical function to operate the arrays. Pandas provided data structures and operations for manipulating numerical tables. Seaborn helps with a high-level interface for drawing on statistical graphs. All these libraries are present in Scikit learn as a package. TensorFlow is used for machine learning applications such as neural networks. Keras is a specific library designed for fast experimentation with neural networks. Normalization is then applied to normalize the distribution and increase the success rate. In this study, the standardization/*z*-score normalization procedure was utilized. Standardization is performed to guarantee that the features are properly normalized.

Data preprocessing is done first, then data is examined for discrepancies or missing values, and then random sampling is done. Sampling creates a one-of-a-kind sampling distribution based on actual facts. The purpose of sampling is to provide a more accurate assessment of the chosen features. After that, the data is normalized.

### 4.2. Feature Selection

The second step is the features selection, and it involves several filter-based methods. The analysis to identify the strongest predictors to address using correlation analysis is followed by recursive feature elimination method. For picking the strongest predictors, this approach proves better than other nonparametric approaches such as the *K*-Nearest Neighbors which would not be able to rank predictors according to their importance.

We advocate the use of a hybrid of correlation-based elimination strategy and recursive feature elimination because this will result in a better selection of optimal features. Even after features are eliminated by correlation, there might still be features that are not very useful; hence, a second step using recursive feature elimination will ensure the right selection of features.

### 4.3. Classification

The third step is classification. In this step, the selected features from the previous step are fed as input to the classification model. Fivefold cross-validation is performed; i.e., 80% percent of the whole data is used in the training phase, and 20% percent is used in the testing phase. The machine learning model then classifies this dataset to detect breast cancer. The details of the machine learning model and classification results are discussed in detail in the section.

## 5. Experimental Evaluation

This section explains the dataset and the tools and technologies used for the development of the EDFBC framework.

### 5.1. Experimental Setup

#### 5.1.1. Dataset

In this study, the WDBC dataset has been utilized and accessed from the UCI library. The Wisconsin Diagnostic Breast Cancer (WDBC) dataset contains 569 samples in total [26]. Target values indicate that the person's tumor is malignant (cancerous) or benign (noncancerous). The WDBC includes the 569 samples distributed between malignant and benign samples. From the total 569 samples, 357 samples are benign and the rest 212 samples of malignant breast cancer cases are present.

#### 5.1.2. Utilized Platforms

Exploratory analysis and data processing are performed in the following environment:

- Python version 3.7
- Numpy (package for multidimensional array processing and indexing)
- Pandas (package for data analysis and manipulation tool, providing easy to use data structures)
- Matplotlib and Seaborn (package provides high-level interfaces for creating attractive and informative statistical graphs)
- Scikit learn libraries for various classification algorithms (machine learning library that provides various algorithms)
- Keras (open-source neural network library, enabling fast experimentation with deep neural networks)
- TensorFlow (symbolic math library used for machine learning applications)

### 5.2. Sampling and Normalization

This section describes the data exploration and preprocessing activities and the valuable insights gathered from an exploratory analysis. The first step that is performed is data preprocessing. The process of data preprocessing including normalization, sampling, and test-train splitting is discussed below.

First, an exploratory analysis of the data was done. The data was visualized to see feature importance, correlation, and the variation in values of different features. Data visualization and exploration are important steps before we input the data into any machine learning algorithm. The WDBC constitutes nine numerical predictors and a binary dependent variable, indicative of the presence of breast cancer.  Table 2 shows the distribution of the WDBC dataset.

The dataset consists of a total of 33 features, out of which there are an “unnamed 32” attribute and an ID attribute that have been removed manually. One of the features is the class tag, and the rest are used for feature selection. Further, we perform data sampling and normalization.

### 5.3. Attribute Selection

The attribute selection analysis is performed to identify the strongest predictors that are addressed using connected analysis followed by a repeated feature elimination method. Other nonparametric supervised learning approaches such as *K*-Nearest Neighbors may not be able to rank the predictors by their importance.

Firstly, the features were eliminated on the base of correlation. The correlated attributes and the selected attributes are summarized in Table 3. The correlation among the 30 attributes is demonstrated through a heat-map analysis shown in Figure 2. The association among the multiple parameters is displayed through different colors. The lighter colors show the high correlation between the two attributes, and the white color shows the high association with a maximum value of 1. On contrary, the darker colors represent the least correlation.

This process reduced the number of features from 30 to 16. To check if the feature selection is correct, the recall value for the chosen features has been calculated. The values obtained from different algorithms were all greater than 90, with the highest recall value of 93.6% with the Random Forest algorithm, and the *f*-score value was 0.95. The recall was computed for the testing dataset.

The second step involved recursive feature elimination (RFE). RFE assigns weights to each feature. Those features that carry the smallest absolute weights are pruned from the present feature set [40]. This process is repeated until the required number of features is reached. 16 features were computed through RFE with an improved recall value of 93.7%. These 16 features were different from the ones computed previously. The Scikit platform provides an algorithm, i.e., the RFECV, which automatically finds the optimal number (and choice) of features required for best scoring. The RFECV algorithm is used to find the best scoring features. The optimal number of features according to the RFECV came out to be 20. However, the best 20 features included correlated features like radius_mean, perimeter_mean, and area_mean together, which did not seem to be very useful.  Figure 3 shows the feature importance of features selected by recursive feature elimination.

The number of features required to optimize the algorithm after the elimination of correlated features was found to be 11. The RFE algorithm is used with fixed 11 features. The selected features were the ones that were appearing most in the solution.  Table 4 shows the value of feature scores for the above 16 features.

### 5.4. Classification

The finalized set of 11 attributes was used for classification by the ML models including Random Forest Classifier, Gradient Boosting Classifier, Support Vector Machines (SVM), Artificial Neural Network, and Multilayer Perception model. Five classification algorithms are used in order to determine the performance of each model with a reduced feature space. Their performance and accuracy are analyzed by cross-validation techniques.

Artificial Neural Networks are mainly divided into two categories based on the way to learn the data and patterns: supervised and unsupervised. In the supervised learning environment, the network is provided with both the input and correct outputs. During the training phase, the network generates its outputs, matched them with the true outputs, and then readjusted the weights to best match the true outputs in an iterative process. On the other hand, in an unsupervised environment, the neural network is provided with the inputs, but without output. The network then finds the pattern between the data and calculates acceptable weights by developing a representation of input stimuli. The input data is clustered, and features that are valuable for the solution are discovered.

Analyzing differing models in the literature, we have utilized the Multilayer Perceptron Model as it provides high generalization ability and has shown encouraging results on standard prediction and classification datasets in the medical field.  Table 5 summarizes the results obtained from the finalized set of 11 attributes used for classification by machine learning models. It also displays the accuracy percentage result of each ML algorithm. The best accuracy of 99.12% is achieved by the MLP model. The best train-test split was determined to be 80-20 (5-fold cross-validation).

## 6. Results and Comparative Analysis

In our approach, we begin with data preprocessing. After checking for discrepancies or missing values, the data is sampled. Random sampling creates a one-of-a-kind sampling distribution based on the data. Normalization is then applied to normalize the distribution and increase the success rate. Standardization/*z*-score normalization is used to ensure good normalization of the features. It is the most commonly used method in machine learning algorithms. In *z*-score normalization, all indicators are converted into a common scale, having a standard deviation of one and an average of zero. This method is preferred over other methods because the average of zero is used. This means that it avoids introducing aggregation distortions. Since the data has no missing value, this method will be beneficial.

As a consequence, a set of 11 characteristics is generated, which is subsequently used as input to classification models. Five classification algorithms are used in order to determine the performance of each with a reduced feature space. Their performance is analyzed, and their accuracies are analyzed. The classification was performed with different test-train splits. The best train-test split was determined to be 80-20 (5-fold cross-validation).

This allows us to select the strongest predictors from the entire feature space. Correlation-based selection and recursive feature removal approaches are then used to choose features [28]. First, the features are analyzed for correlation. The highly correlated features are set aside, and one of them is chosen, so that if three features are highly connected, one of them is chosen. The data is then subjected to recursive feature elimination (RFE) in order to extract the best features. The comparison of machine learning algorithms on Wisconsin Breast Cancer dataset is shown in Table 6.

### 6.1. Application of BCAD Framework on Different Datasets

Our proposed approach was targeted at improving the overall classification process by prosing a framework comprising of data handing and filter-based feature selection methods and testing the performance over different train and test splits. By reducing the number of features, the performance of the model is optimized and the overall generalizability of the model is optimized. The overall training time is reduced and the generalizability of the model is increased. Both accuracy and generalization have been leveraged through correct and better feature selection. The computational complexity is reduced.

We advocated the use of correlation-based elimination strategy, followed by recursive feature elimination because this resulted in a better selection of optimal features. Even after features are eliminated by correlation, there might still be features that are not very useful; hence, a second step using recursive feature elimination ensures the right selection of features.

We have applied our framework to additional two datasets of breast cancer that include the Wisconsin Original Dataset for Breast Cancer (WOBC) [29] and the Wisconsin Prognostic Dataset for Breast Cancer (WPBC) [30] and recorded the results. The WPBC dataset consists of features computed from fine images of the breast mass of patients. The standard error, mean value, and largest mean (worst case-mean of the three largest values) are computed for these features, and as a result, 30 features are obtained that are listed in the dataset. The target attribute is the outcome (class label). All attributes except the attribute ID can be used as predicted variables, whose values can be used for determining the results. The WOBC dataset consists of samples collected periodically. There are a total of 10 features and one class label. The data are grouped in chronological order from groups of data recorded from January 1989 to November 1991.

We have applied our approach by selecting careful features and data handling on the WOBC and WPBC datasets. The proposed solution improves the overall classification process. The accuracy of classification is affected greatly by careful feature selection. Overall classification process, the classification accuracy, and the training time are improved by careful feature selection.

The comparison of our proposed model with various ML-based approaches developed and used by researchers on WOBC and WPBC is represented in Table 7.

Both datasets, WOBC and WPC, were subjected to our framework, and the results were recorded. First, standardization is carried out to verify that features are properly normalized, and then feature selection is carried out. Filter-based feature selection procedures like correlation analysis and recursive feature reduction are used to find the strongest predictors. Our suggested EDFBC framework clearly outperforms state-of-the-art techniques. Choosing the right features improves the whole classification process, increasing accuracy and minimizing the time of training data.

## 7. Conclusion

In this paper, a new framework has been proposed for the detection of breast cancer. The proposed framework includes three main stages, i.e., data preprocessing, feature selection, and classification. The classification experiments were performed using SVM, Random Forest, Gradient Boosting, Artificial Neural Network, and Multilayer Perceptron Model on the WDBC dataset. With a 99.12% accuracy, the Multilayer Perceptron Model outperformed all other models under investigation. In addition, the obtained results have also been compared with the experiments performed on the WPBC and WOBC datasets. The results indicate the exceptional performance of the proposed framework with the MLP model and the WDBC dataset when compared with other state-of-the-art approaches. In the future, our plan is to use a random neural network along with MLP for higher accuracy and precision. Also, we will validate the proposed model on other datasets as well.

## Figures and Tables

**Figure 1:** Breast Cancer Diagnostic (BCAD) framework.

**Figure 2:** Heatmap analysis of features.

**Figure 3:** Feature importance.

**Table 1:** Comparison of machine learning algorithms on the WDBC dataset.

Author	Year	Features	Classifier	Accuracy achieved (%)
Aryal & Paudel [36]	2020	30	Gradient Boosting	98.88%
Ahmet Saygili [37]	2018	24	Random Forest	98.77%
Dubey et al. [38]	2016	—	*K*-means clustering	92.00%
Salama et al. [39]	2012	30	SMO	97.71%

**Table 2:** Wisconsin (Diagnostic) Breast Cancer dataset.

Total samples	569
Malignant	357
Benign	212

**Table 3:** Selected attributes based on correlation.

Correlated attributes	Selected attribute
compactness_mean, concavity_mean, concave points_mean	concavity_mean
radius_se, perimeter_se, area_worst	area_se
compactness_worst, concavity_worst, concave points_worst	concavity_worst
compactness_se, concavity_se, concave points_se	concavity_se
texture_mean, texture_worst	texture_mean
area_worst, area_mean	area_mean

**Table 4:** Feature importance scores of selected features.

Attribute	Scores
Area_mean	0.213700
Concavity_mean	0.188830
Area_se	0.165063
Concavity_worse	0.143952
Concavity_se	0.058901
Smoothness_worst	0.047903
Fractal_dimension_se	0.030430
Texture_mean	0.025588
Smoothness_mean	0.025035
Symmetry_worst	0.023982
Smoothness_se	0.021418
Texture_se	0.015029
Symmetry_mean	0.014530
Fractal_dimension_worst	0.013285
Fractal_dimension_mean	0.006309
Symmetry_se	0.006046

**Table 5:** Classification accuracy.

Machine learning method	Ratio (training: testing)		
	60 : 40	70 : 30	80 : 20
	Accuracy		
Random Forests	95.40%	96.67%	98.07%
ANN	93.02%	85.53%	97.35%
Gradient Boosting	94.56%	95.70%	97.07%
SVM	97.55%	97.21%	97.76%
MLP	98.11%	98.99%	99.12%

**Table 6:** Comparison of machine learning algorithms on Wisconsin Breast Cancer dataset.

Author	Year	Dataset	Imbalance handling	Feature selection	Features	Classifier	Validation type	Accuracy achieved (%)
Aryal & Paudel [37]	2020	WDBC	—	—	30	Gradient Boosting	10-fold	98.88%
Ahmet Saygili [38]	2018	WDBC	—	Gain Ratio	24	Random Forest	10-fold	98.77%
Dubey et al. [39]	2016	WDBC	—	—	—	*K*-means clustering	—	92.00%
Salama et al. [41]	2016	WDBC	—	—	30	SMO	10-fold	97.71%
Our approach	2020	WDBC	Normalization by standardization	Correlation-based selection & RFE	11	MLP	5-fold	99.12%

**Table 7:** Comparison of machine learning algorithms on Wisconsin Breast Cancer dataset.

Author	Year	Dataset	Imbalance handling	Feature selection	Features	Classifier	Validation type	Accuracy achieved %
Wisconsin original breast cancer dataset (WOBC) [23]								
Salama et al. [41]	2012	WOBC	—	Chi-square & PCA	10	J48 & MLP	10-fold	97.28%
Hamsagayathri & Sampath [42]	2017	WOBC	—	Feature ranking	—	Random Forest	10-fold	96.70%
Our approach	2020	WOBC	Normalization by standardization	Correlation based selection & RFE	8	MLP	5-fold	98.20%
Wisconsin Prognostic breast cancer data (WPBC) [24]								
Tintu and Paulin [43]	2013	WPBC	Manual removal of instances	Feature ranking	—	Fuzzy *C*-means clustering	4-fold	97.13%
Khan et al. [44]	2013	WPBC	—	YAGGA	19	Linear regression	10-fold	84.34%
Our approach	2020	WPBC	Normalization by standardization	Correlation-based selection and RFE	16	MLP	5-fold	98.33%

## Data Availability

The Wisconsin Diagnostic Breast Cancer dataset is available at https://archive.ics.uci.edu/ml/datasets/breast+cancer+wisconsin+(diagnostic%7d}. The SEER Breast Cancer dataset is available at https://ieee-dataport.org/open-access/seer-breast-cancer-data.
